The article "Exosomal miR‐1255b‐5p targets human telomerase reverse transcriptase in colorectal cancer cells to suppress epithelial‐to‐mesenchymal transition" was retracted in 2023. Reasons: duplicated images; original data or images not available.

# Exosomal miR‐1255b‐5p targets human telomerase reverse transcriptase in colorectal cancer cells to suppress epithelial‐to‐mesenchymal transition

**DOI:** 10.1002/1878-0261.12765

**Published:** 2020-08-19

**Authors:** Xue Zhang, Jian Bai, Hang Yin, Long Long, Zhewen Zheng, Qingqing Wang, Fengxia Chen, Xiaoyan Yu, Yunfeng Zhou

**Affiliations:** ^1^ Department of Radiation Oncology and Medical Oncology Zhongnan Hospital of Wuhan University Wuhan China; ^2^ Hubei Key Laboratory of Tumor Biological Behaviors Wuhan China; ^3^ Hubei Cancer Clinical Study Center Wuhan China; ^4^ Department of Gastrointestinal Surgery & Department of Gastric and Colorectal Surgical Oncology Zhongnan Hospital of Wuhan University Wuhan China

**Keywords:** epithelia‐to‐mesenchymal transition, exosome, hTERT, microenvironment, microRNA

## Abstract

Cancer cells undergo epithelial‐to‐mesenchymal transition (EMT) in response to hypoxia. Exosomes produced in tumor microenvironments carry microRNAs (miRNAs) that affect proliferation, metastasis, and EMT. Hypoxic regulation of EMT is associated with telomerase content and stability, but the underlying mechanisms remain unclear. We identified a targeting relationship between tumor‐suppressing miR‐1255b‐5p and human telomerase reverse transcriptase (hTERT) via clinical screening of serum samples in colorectal cancer (CRC) patients. EMT suppression via exosomal miR‐1255b‐5p delivery was investigated by assessing hTERT expression, Wnt/β‐catenin signaling, and telomerase activity. We revealed that hypoxia directly affected exosomal miR‐1255b‐5p content, the delivery of which between CRC cells significantly impacted cell invasion, EMT‐related protein expression, and telomerase stability. Specifically, miR‐1255b‐5p suppressed EMT by inhibiting Wnt/β‐catenin activation via hTERT inhibition. Hypoxia reduced exosomal miR‐1255b‐5p secretion by CRC cells, thereby increasing hTERT expression to enhance EMT and telomerase activity. In a mouse CRC model, hypoxic exosomes containing overexpressed miR‐1255b‐5p attenuated EMT, tumor progression, and liver metastasis. Our results suggest the antitumor role of miR‐1255b‐5p and its involvement in the regulation of hTERT‐mediated EMT. We propose that miRNA‐targeted regulation of telomerase is a promising therapeutic strategy for future CRC treatment.

## Graphical abstract

Cancer cells undergo epithelial‐to‐mesenchymal transition (EMT) in response to hypoxia. Tumor‐derived exosomes carry microRNAs (miRNA) that affect metastasis and EMT. We identified a targeting relationship between tumor‐derived exosomal miR‐1255b‐5p and human telomerase reverse transcriptase in association with EMT and telomerase stability. We propose miRNA‐targeted regulation of telomerase as a promising strategy for CRC treatment.

The article "Exosomal miR‐1255b‐5p targets human telomerase reverse transcriptase in colorectal cancer cells to suppress epithelial‐to‐mesenchymal transition" was retracted in 2023. Reasons: duplicated images; original data or images not available.

**Abbreviations**
ANOVA: analysis of variance
CCK‐8: cell‐counting kit‐8
CEA: carcinoembryonic antigen
CRC: colorectal cancer
EMT: epithelial‐to‐mesenchymal transition
GST: glutathione S transferase
H&E: hematoxylin/eosin
HIF‐1: hypoxia‐inducible factor‐1
hTERT: human telomerase reverse transcriptase
inh: inhibitor
LVI: lymphovascular invasion
mim: mimic
miRNA: microRNA
MUT: mutant
nc: negative control
PNI: perineural invasion
qRT‐PCR: quantitative reverse transcription polymerase chain reaction
RISC: RNA‐induced silencing complex
TEM: transmission electron microscopy
WT: wild‐type
ZEB1: zinc finger E‐box‐binding homeobox 1
CA 19‐9: carbohydrate antigen 19–9

## 1 Introduction

Among the most prevalent malignancies worldwide, colorectal cancer (CRC) is one of the most deadly and difficult to treat and manage, with 97 220 new cases and causing approximately 50 630 related deaths in the United States in 2018 [1]. Metastasis is the main cause of CRC‐related deaths, and one of the underlying mechanisms of metastasis is pre‐invasive epithelial‐to‐mesenchymal transition (EMT), which is associated with poor prognosis. EMT is the process through which cancer cells acquire invasive mesenchymal cell‐like properties, resulting in metastasis from the primary tumor site to adjacent tissues or even distal sites and ultimately leading to resistance to therapeutic intervention [2]. The occurrence of EMT has been linked to diverse factors, one of which is the deficiency in oxygen, or hypoxia. In most solid tumors, when tumor growth reaches a certain extent, vascular growth becomes defective and restricted because of poor blood supply, causing the cancer cells to be present in a hypoxic state [3, 4]. In cells exposed to a hypoxic environment, the transcription factor hypoxia‐inducible factor‐1 (HIF‐1) is activated to promote the release of angiogenic factors [4] and the expression of genes such as glucose transporters and glycolytic enzymes, inducing cell proliferation and invasion [5, 6]. In turn, hypoxia provides a favorable microenvironment for the exacerbation of cancer cell growth and tumor metastasis.

MicroRNA (miRNA)‐based therapy has recently emerged as a highlighted trend in cancer treatment and has demonstrated remarkable potential in the development of targeted therapy. These short, noncoding RNAs are composed of 18–25 nucleotides and mediate the expression of their target genes via upregulation (activation) or downregulation (inactivation). A number of miRNAs have been shown to be associated with EMT in CRC. miR‐140 was proven to inhibit EMT by targeting Smad3, in turn suppressing CRC tumor formation and metastasis [7]. Members of the miR‐34 family also suppress CRC progression by negatively regulating EMT [8]. Numerous cytokines, transcription factors, matrix metalloproteinases, and miRNAs are involved in the development of EMT in tumor cells under hypoxic/anoxic conditions. These biologically active molecules with regulatory effects are transported by extracellular microvesicles, known as exosomes, produced by tumor cells. Under hypoxic conditions, cancer cell‐derived exosomes are abundantly and rapidly released into the tumor microenvironment and have multiple roles in tumor growth and metastasis, including angiogenesis and immune regulation [9, 10]. Studies have reported that exosomes produced by colon cancer cells in hypoxic environments may have a promoting effect on cell invasion and metastasis [11], but the specific functions and potential mechanisms remain to be elucidated.

The article "Exosomal miR‐1255b‐5p targets human telomerase reverse transcriptase in colorectal cancer cells to suppress epithelial‐to‐mesenchymal transition" was retracted in 2023. Reasons: duplicated images; original data or images not available.

Telomerase is an enzyme that maintains and lengthens telomere ends, and the telomerase complex is composed of telomerase RNA, dyskerin, and telomerase reverse transcriptase (TERT) [12]. While telomerase is normally absent in somatic cells, it is active in stem cells and cancer cells. Deficiencies in telomerase (and TERT) have been linked to aging‐related conditions [13], whereas the overexpression of TERT is associated with cancer and tumor progression [14]. Human TERT (hTERT) has been shown to form a complex with zinc finger E‐box‐binding homeobox 1 (ZEB1), and this complex inhibits epithelial cadherin (E‐cadherin) expression by recruiting BRG1 and binding to the promoter region of the E‐cadherin gene, thereby promoting EMT [15, 16]. Under hypoxic conditions, hTERT is further upregulated in tumor cells to enhance their survival ability in hypoxic environments [17, 18]. hTERT reportedly regulates EMT in gastric cancer cells through transforming growth factor‐β and β‐catenin signaling [19], whereas Wnt signaling mediates this effect in oral squamous cell carcinoma [20]. However, the regulation of EMT by hTERT under hypoxia in CRC cells has not been investigated.

We hypothesized that in hypoxic environments, CRC cells produce a large number of exosomes that are released into the tumor environment, and these exosomes carry miRNAs associated with hypoxia‐induced EMT. This study was carried out by considering clinical, *in vitro*, and *in vivo* aspects, with the aim of gaining an overall insight into the effect of exosomal miRNA delivery on EMT‐associated CRC metastasis. We identified the key miRNAs involved in this phenomenon and elucidated the role of hTERT therein, in turn clarifying the underlying participation of the Wnt/β‐catenin pathway in the mechanisms that mediate this process.

The article "Exosomal miR‐1255b‐5p targets human telomerase reverse transcriptase in colorectal cancer cells to suppress epithelial‐to‐mesenchymal transition" was retracted in 2023. Reasons: duplicated images; original data or images not available.

## 2 Materials and methods

### 2.1 Patients and serum sample for preliminary bioinformatic screening

Primary CRC serum samples were obtained from 70 patients diagnosed with primary CRC at Zhongnan Hospital of Wuhan University (Wuhan, China). All samples were collected with informed consent from the patients, and all related procedures were performed with the approval of the internal review and ethics boards of Zhongnan Hospital of Wuhan University. All study methodologies conformed to the standards set by the Declaration of Helsinki. Preliminary miRNA screening was performed using the Gene Expression Omnibus dataset GSE39833 (miRNA profiles of serum exosomes in healthy controls and CRC patients). Among the miRNAs showing differential expression, those with binding sites to the 3′UTR of hTERT were identified using the TargetScan web server (http://www.targetscan.org/vert_72/). The expression of the identified miRNAs was evaluated in exosomes isolated from the previously collected serum samples.

### 2.2 Cell culture and treatment

Human CRC cell lines SW480, HCT116, LOVO, HT29, and a normal fetal colon cell line (FHC) were obtained from the cell bank of the Chinese Academy of Sciences (Shanghai, China). SW480 cells were cultured in L15 medium (41300‐039; Gibco, Waltham, MA, USA), HCT116 cells were cultured in McCoy's 5A medium (16600‐082; Gibco), LOVO cells were cultured in F12K medium (21127‐022; Gibco), HT29 cells were cultured in McCoy's 5A medium, and FHCs were cultured in Dulbecco's modified Eagle's medium/F‐12 (SH30023.01; Hyclone, Carlsbad, CA, USA). All media were supplemented with 10% FBS (10270‐106; Gibco). To achieve a hypoxic microenvironment, cells were cultured in an AnaeroPack hypoxia kit (Genel, Shanghai, China) according to the manufacturer's instructions. For the subsequent experiments, normoxic conditions were defined as 21% oxygen and 5% CO_2_, whereas hypoxic conditions were defined as 1% oxygen, 5% CO_2_, and 94% N_2_. Normoxic and hypoxic culture were performed for 24 and 48 h, respectively, before the cells were subjected to subsequent experiments.

### 2.3 Overexpression and silencing of miR‐1255b‐5p and hTERT

To overexpress or silence miR‐1255b‐5p, CRC cells were transfected with commercially synthesized mimics and inhibitors of miR‐1255b‐5p (GenePharma, Shanghai, China). Transfection was performed by incubating cells with miR‐1255b‐5p mimics or inhibitors at 1 nm for 6 h, after which the transfection efficiency was measured. For hTERT interference, pSICOR interference vectors were purchased from Addgene (Watertown, MA, USA). The hTERT interference fragment (sequence: GGAATCAGCAGGAGGAGATCT) was inserted into the pSICOR vector with XhoI and BamHI restriction sites to produce si‐hTERT. CRC cells were transfected with si‐hTERT or its corresponding negative control (NC) plasmid (nc‐hTERT) using Lipofectamine 2000 (11668‐027; Invitrogen, Carlsbad, CA, USA) according to the manufacturer's instruction.

The article "Exosomal miR‐1255b‐5p targets human telomerase reverse transcriptase in colorectal cancer cells to suppress epithelial‐to‐mesenchymal transition" was retracted in 2023. Reasons: duplicated images; original data or images not available.

### 2.4 Exosome isolation and characterization

Exosomes were isolated from either the serum of clinical CRC patients (or healthy individuals) or SW480 cells that were cultured in normoxic or hypoxic conditions for 24 h. Serum or cell samples were centrifuged for 10 min at 500 ***g***, and the supernatant was collected and centrifuged for 20 min at 2000 ***g***. The supernatant was then ultracentrifuged (Optima L‐100 XP; Beckman Coulter, Brea, CA, USA) for 70 min at 100 000 ***g***, and the precipitate was resuspended in 20 mL of PBS. The mixture was again ultracentrifuged for 70 min at 100 000 g, and the precipitate was resuspended in PBS at a ratio of 1 : 20. After 20 min of centrifugation at 2000 ***g***, the supernatant was collected and subjected to 40% sucrose density gradient purification at 100 000 g for 70 min. The supernatant underwent a final round of ultracentrifugation for 70 min at 100 000 g, resulting in precipitate containing the isolated exosomes. To visualize exosomes using transmission electron microscopy (TEM), the exosomes were fixed in 2% glutaraldehyde in 0.1 m PBS (pH = 7.4). The fixed exosomes were dropped onto a nickel mesh and washed with PBS after 30 min. Then, 1% glutaraldehyde was dropped onto the mesh and incubated for 5 min, and the specimen was washed with double‐distilled water several times. Filtered 4% uranyl acetate was then dropped onto the specimen, and after 5 min, excess liquid was removed using filter paper and the dried specimen was subjected to TEM analysis (HT7700; Hitachi, Research Center for Medicine and Structural Biology, Wuhan University) at the Research Center for Medicine and Structural Biology of Wuhan University. All subsequent functional assays involving exosomes were performed using 10 mg·mL^−1^ purified exosomes. Exosome endocytosis was evaluated via PKH67 labeling using a PKH67 Green Fluorescent Cell Linker Midi Kit (MIDI67‐1KT; Sigma‐Aldrich, St. Louis, MO, USA) prior to cellular uptake. Isolated exosomes (10 μg) were mixed with 1 mL of diluent reagent (provided in the kit) and 4 μL of PKH67 solution. After 4 min of incubation, 2 mL of 0.5% bovine serum albumin in PBS was added to remove the excess dye. The PKH67‐labeled exosomes were ultracentrifuged at 100 000 ***g*** at 4 °C for 70 min and resuspended in 100 μL of PBS. To assess exosome uptake, HCT116 cells were seeded onto a 24‐well plate at 1 × 10^4^ cells per well and cultured for 12 h at 37 °C in an atmosphere containing 5% CO_2_. Then, 10 μg of PKH67‐labeled exosomes was added to each well and the cells were incubated at 37 °C in 5% CO_2_. After 2, 24, or 48 h, the cells were fixed for 20 min with 4% paraformaldehyde and the nuclei were stained with Hoechst 33258. The cells were then observed using a fluorescence microscope, and green fluorescence represents the uptake of PKH67‐labeled exosomes.

The article "Exosomal miR‐1255b‐5p targets human telomerase reverse transcriptase in colorectal cancer cells to suppress epithelial‐to‐mesenchymal transition" was retracted in 2023. Reasons: duplicated images; original data or images not available.

### 2.5 Scratch assay

Cells were seeded in 6‐well plates at 1 × 10^6^ cells per well, cultured overnight, and subjected to treatment accordingly. A scratch was made in the cell monolayer using a pipette tip placed perpendicular to the bottom surface of the well. After the scratch was made, the wells were washed with PBS, and serum‐free medium was added to each well. Cell culture continued at 37 °C in an incubator containing 5% CO_2_. Images of gap closure were acquired using an optical microscope at 0, 24, and 48 h after scratching.

### 2.6 Cell‐counting kit‐8 (CCK‐8) assay

Cells were seeded in a 96‐well plate at 5 × 10^3^ cells per well with 180 μL of medium in each well. The plate was incubated overnight at 37 °C in 5% CO_2_, and the medium was replaced. Cells were treated accordingly and cultured for 24 or 48 h. Thereafter, 10 μL of CCK‐8 solution was added to each well, and the cells were further incubated for 4 h at 37 °C. The absorbance of the wells was measured using a plate reader at 450 nm (Multiskan FC, Thermo Fisher Scientific, Waltham, MA, USA), and the degree of cell proliferation is represented by the relative optical intensity.

### 2.7 Transwell invasion assay

A Transwell assay was performed to evaluate the invasion of cells subjected to various treatments. Prior to the experiment, Transwell inserts (Corning Inc., Corning, NY, USA) were placed into the wells of a 24‐well plate and coated with 80 μL of Matrigel (354230; BD Biosciences, Franklin Lakes, NJ, USA) at 37 °C for 30 min. Treated cells were cultured for 24 h in serum‐free medium, trypsinized, and seeded into the top chamber of the coated Transwell inserts at 1 × 10^5^ cells per mL (500 μL). In the bottom chamber, 750 μL of medium containing 10% FBS was added. The plate was incubated at 37 °C for the indicated amount of time, after which the medium was removed and the cells were fixed with 1 mL of 4% paraformaldehyde in each well for 10 min at room temperature. The fixative was removed, the cells were washed once with PBS, and 1 mL of 0.5% crystal violet solution (PAB180004, Bio‐Swamp) was added to each well. After 30 min of staining, the cells were washed three times with PBS. Cells that have invaded to the bottom chamber of the Transwell inserts were imaged using an optical microscope at 200×. Stained cells in each field of view were counted and quantified using imagej (National Institutes of Health, Bethesda, MD, USA).

The article "Exosomal miR‐1255b‐5p targets human telomerase reverse transcriptase in colorectal cancer cells to suppress epithelial‐to‐mesenchymal transition" was retracted in 2023. Reasons: duplicated images; original data or images not available.

### 2.8 Quantitative reverse transcription polymerase chain reaction (qRT‐PCR)

RNA was extracted using TRIzol (15596026; Ambion, Inc., Foster City, CA, USA) and reverse‐transcribed into cDNA using the RevertAid First Strand cDNA Synthesis Kit (K1622; Thermo Scientific). qRT‐PCR was carried out using the SYBR Green PCR kit (KM4101; KAPA Biosystems, Wilmington, MA, USA) with the following primer sequences: hTERT F, 5′‐CAGGCACAACGAACGC‐3′, R, 5′‐TCCTCACGCAGACGGT‐3′; HIF‐1α F, 5′‐ATCTCCATCTCCTACCC‐3′, R, 5′‐TGACTCCTTTTCCTGC‐3′; E‐cadherin F, 5′‐GCTCACATTTCCCAACTC‐3′, R, 5′‐TGCTGTAGAAAACCTTGC‐3′; vimentin F, 5′‐TGAACGCAAAGTGGAATC‐3′, R, 5′‐AGGTCAGGCTTGGAAACA‐3′; β‐actin F, 5′‐ACACTGTGCCCATCTACG‐3′, R, 5′‐TGTCACGCACGATTTCC‐3′. Stem‐loop qRT‐PCR was performed for miR‐1182, miR‐1255b‐5p, and miR‐197‐3p using the following primers: miR‐1182 stem‐loop primer, CTCAACTGGTGTCGTGGAGTCGGCAATTCAGTTGAGGTCACATC; miR‐1182 forward, GGGGAGGGTCTTGGGAGG; miR‐1182 reverse, AACTGGTGTCGTGGAGTCGGC; miR‐1255b‐5p stem‐loop primer, CTCAACTGGTGTCGTGGAGTCGGCAATTCAGTTGAGAACCACTT; miR1255b‐5p forward, GGGCGGATGAGCAAAGA; miR1255b‐5p reverse, AACTGGTGTCGTGGAGTCGGC; miR‐197‐3p stem‐loop primer, CTCAACTGGTGTCGTGGAGTCGGCAATTCAGTTGAGGCTGGGTG; miR‐197‐3p forward, GGGTTCACCACCTTCTC; miR‐197‐3p reverse, AACTGGTGTCGTGGAGTCGGC; U6 forward, CTCGCTTCGGCAGCACA; U6 reverse, AACGCTTCACGAATTTGCGT. The experimental conditions were as follows: 95 °C for 3 min (initial denaturation); 39 cycles of denaturation at 95 °C for 5 s, annealing at 56 °C for 10 s, and extension at 72 °C for 25 s; and 65 °C for 5 s and 95 °C for 50 s (final extension). Data acquisition was carried out using the QuantStudio™ 6 Flex Real‐Time PCR System (Applied Biosystems, Foster City, CA, USA) and analyzed with the $2^{‐\Delta \Delta C_{t}}$ method.

### 2.9 Evaluation of RNA stability

HCT116 cells were seeded into the wells of a 6‐well plate and transfected with miR‐1255b‐5p mimics or its corresponding NC as described in Section 2.3. After 48 h of transfection, actinomycin D (abs810015; Absin, Shanghai, China) as added to each well at 5 μg·mL^−1^. RNA was extracted from the cells at 0, 2, 4, 8, and 16 after the addition of actinomycin D, and the mRNA expression of FOXO4 was evaluated by PCR as described in Section 2.8.

### 2.10 Western blot

Lysates from cell or tissue samples were harvested using radioimmunoprecipitation assay buffer supplemented with protease and phosphate inhibitors. Western blot was performed on polyvinylidene fluoride membranes (IPVH00010; Millipore, Burlington, MA, USA) using 20 μg of protein in denaturing conditions for CD63 (ab217345; Abcam, Cambridge, UK), CD81 (ab103201; Abcam), TSG101 (ab30871; Abcam), hTERT (rabbit, 1 : 1000, ab230527; Abcam), HIF‐1α (1 : 1000, PAB37598, Bio‐Swamp), E‐cadherin (1 : 1000, PAB30714, Bio‐Swamp), vimentin (1 : 1000, PAB30692, Bio‐Swamp), Wnt1 (rabbit, 1 : 1000, PAB40578, Bio‐Swamp), β‐catenin (rabbit, 1 : 4000, ab6302; Abcam), and β‐actin (mouse, 1 : 5000, 66009‐1‐Ig; Proteintech, Chicago, IL, USA). Primary antibody incubation was performed overnight at 4 °C, after which the membranes were incubated with goat anti‐rabbit IgG (1 : 10 000, PAB160011, Bio‐Swamp) or goat anti‐mouse IgG (1 : 10 000, PAB160009, Bio‐Swamp) secondary antibodies for 1 h at 4 °C in the dark. The membranes were then immersed in an enhanced chemiluminescence reagent (WBKLS0010; Millipore), and protein bands were visualized using a Tanon‐5200 automatic analyzer (Tanon, Shanghai, China) and a Bio‐Rad ChemiDoc XRS + System (Bio‐Rad, Hercules, CA, USA). Band gray values were obtained using Tanon gis software or bio‐rad image analysis software. All protein expression was normalized to that of β‐actin as a loading control.

The article "Exosomal miR‐1255b‐5p targets human telomerase reverse transcriptase in colorectal cancer cells to suppress epithelial‐to‐mesenchymal transition" was retracted in 2023. Reasons: duplicated images; original data or images not available.

### 2.11 Assessment of telomerase content

Telomerase content was evaluated using an enzyme‐linked immunosorbent assay kit for human telomerase (HM11275; Bio‐Swamp) following the manufacturer's instructions. For the detection of telomere length, DNA was first extracted using a reagent kit (DP304‐02; Tiangen, Hangzhou, China). The DNA was mixed with primers for telomeres (270 nm for TEL1; 900 nm for TEL2) and the single‐copy gene 36B4 (300 nm for 36B4u; 500 nm for 36B4d) as a reference, at a total volume of 5 μL, and qRT‐PCR was performed. The primers were TEL1, 5′‐GGTTTTTGA[GGGTGA]_4_GGGT‐3′; TEL2, 5′‐TCCCGACTAT[CCCTAT]_4_CCCTA‐3′; 36B4u, 5′‐CAGCAAGTGGGAAGGTGTAATCC‐3′; and 36B4d, 5′‐CCCATTCTATCATCAACGGGTACAA‐3′. Telomere amplification was performed at 50 °C for 2 min and 30 cycles of 95 °C for 15 s and 54 °C for 2 s. Single‐copy gene amplification was performed at 50 °C for 2 min, 95 °C for 2 min, and 35 cycles of 95 °C for 15 s and 58 °C for 60 s. Data acquisition was carried out using the QuantStudio™ 6 Flex Real‐Time PCR System (Applied Biosystems) and analyzed with the $2^{‐\Delta \Delta C_{t}}$ method.

### 2.12 Dual‐luciferase activity assay

The starBase V2.0 web site was employed to screen for miRNAs that bind to the 3′UTR of hTERT, and seven‐base binding sites to miR‐1255b‐5p were identified at three regions (1278–1284 bp, 1309–1315 bp, and 1420–1427 bp; GenBank AB085628.1, Ensembl ENSG00000164362) of the hTERT promoter. Reporter plasmids were constructed using pmirGLO plasmids (Addgene) according to the manufacturer's instructions. Wild‐type (WT) and mutant (MUT) 3′UTR segments were prepared as follows: hTERT 1278–1284 WT, 5′‐CTAGCACAGGAGGCTTCAGGGTGGGGCTGGTGATGCTCTCTCATCCTCTTATCATCTCCCAGTCTCATCT‐3′, MUT, 5′‐CTAGCACAGGAGGCTTCAGGGTGGGGCTGGTGATGCTCTCATCCTCTCTTATCATCTCCCAGTCTCATCT ‐3′; hTERT 1309–1315 WT, 5′‐CTAGCTCTTATCATCTCCCAGTCTCATCTCTCATCCTCTTATCATCTCCCAGTCTCATCTGTCTTCCTCT‐3′, MUT, 5′‐CTAGCTCTTATCATCTCCCAGTCTCATCTCATCCTCTCTTATCATCTCCCAGTCTCATCTGTCTTCCTCT ‐3′; hTERT 1420–1427 WT, 5′‐CTAGCCTCATCTCTTATCCTCTTATCTCCTAGTCTCATCCAGACTTACCTCCCAGGGCGGGTGCCAGGCT‐3′, MUT, 5′‐CTAGCCTCATCTCTTATCCTCTTATCTCCTAGTCATCCTCAGACTTACCTCCCAGGGCGGGTGCCAGGCT‐3′. A dual‐luciferase activity kit (LucPair™ Duo‐Luciferase Assay Kit, LF001; GeneCopoeia, Rockville, MD, USA) was employed to detect the signal of firefly luciferase and renilla luciferase using a Glo‐MAX 20/20 analyzer.

The article "Exosomal miR‐1255b‐5p targets human telomerase reverse transcriptase in colorectal cancer cells to suppress epithelial‐to‐mesenchymal transition" was retracted in 2023. Reasons: duplicated images; original data or images not available.

### 2.13 Glutathione S transferase (GST) pull‐down

Recombinant plasmids encoding hTERT and GST were transformed into the BL21 (DE3) strain to produce fusion GST‐tagged hTERT protein (GST‐hTERT). The base sequence encoding BRG1 was cloned into a eukaryotic expression vector encoding a tagged protein (myc‐tag) for 48 h to obtain fusion BRG1 protein. For the GST pull‐down assay, GST‐hTERT was cooled on ice and mixed with 50 μL of GST MagBeads (L00327; GenScript, Piscataway, NJ, USA) and 800 μL of 1% Triton X‐100 in PBS for 1 h at 4 °C. The beads were then washed three times with 1% Triton X‐100 and three times with PBS. The fusion BRG1 protein was mixed with GST‐hTERT at 4 °C and rotated to ensure maximal contact between the proteins. Thereafter, the bound proteins were collected using 40 μL of 5 × loading buffer and boiled for 3 min. After ultracentrifugation, binding between BRG1 and hTERT was detected by western blot using an antibody against myc‐Tag (rabbit, 1 : 1000, ab39688; Abcam).

### 2.14 Nude mouse xenograft model of CRC

All animal experiments were performed in accordance with the Guidelines for Animal Care and Use of the Model Animal Research Institute at Wuhan Myhalic Biotechnology Co., Ltd. and have been approved by the institutional review board (approval number HLK‐20181031‐01). Fifty male BALB/c nude mice (specific‐pathogen‐free, 4 weeks old, 16–20 g, *n* = 10 per group) were obtained from Charles River Laboratories (Beijing, China; permit number: 11400700344179). The animals were housed in an environment with controlled temperature at 22–26 °C and relative humidity of 50–60%, in a 12/12‐h light/dark cycle. To establish the *in vivo* CRC xenograft model, the experimental mice were first anesthetized using sodium pentobarbital (P3761; Sigma‐Aldrich). HCT116 cells (200 μL, 1 × 10^6^ cells per mL) were injected subcutaneously in the right axillary region of each mouse. When the tumor volume reached 50–60 mm^3^, each mouse was treated once with 10 μg of exosomes via tail vein injection. The weight of each mouse and the length (L) and width (W) of the tumor was measured every other day. Tumor volume was calculated as (L × W^2^)/2. On day 21, the mice were sacrificed via cervical dislocation, and the weight of the tumors was measured.

The article "Exosomal miR‐1255b‐5p targets human telomerase reverse transcriptase in colorectal cancer cells to suppress epithelial‐to‐mesenchymal transition" was retracted in 2023. Reasons: duplicated images; original data or images not available.

### 2.15 Hematoxylin/eosin (H&E) and immunohistochemical staining

Tumor and liver tissues were cut into small pieces of ~ 1.5 cm × 1.5 cm × 0.3 cm and fixed in 10% formalin for 2 days. They were then dehydrated and embedded in paraffin wax using conventional methods. Before sectioning, the tissue blocks were cooled at −20 °C for several minutes. Sections were obtained at a thickness of 4 μm and placed on microscopic slides. For H&E staining, the tissue sections were deparaffinized and washed with water for 2 min. The sections were then stained with hematoxylin (PAB180015, Bio‐Swamp) for 3 min, washed, and immersed in 1% hydrochloric acid for 1 min. Bluing was performed for 1 min using a solution of 1 g of lithium carbonate (20022818; Sinopharm Chemical Reagent Co., Ltd., Shanghai, China) in 100 mL of deionized water, after which the tissue sections were washed with water for 3 min and immersed in 0.5% eosin solution (PAB180016; Bio‐Swamp) for 3 min. The samples were washed for 10 s with distilled water, 15 s with 80% EtOH, 15 s with 95% EtOH, 3 min with anhydrous EtOH, and twice with xylene for 5 min each. After the sections were sealed with neutral balsam mounting medium, images were acquired using an optical microscope and analyzed using Leica Application Suite. For immunohistochemical staining, tissue sections were heated for 1 h at 65 °C and immersed twice in xylene for 15 min each for deparaffinization. Then, the sections were soaked in a series of EtOH with decreasing concentration (100%, 95%, 85%, and 75%) for 5 min at each concentration and washed with tap water for 10 min. Antigen retrieval was performed using 0.01 m sodium citrate buffer for 15 min at 125 °C and a pressure of 103 kPa. After cooling, the sections were washed three times with PBS for 3 min each, and endogenous peroxidase removal was performed in 3% H_2_O_2_ for 10 min. The sections were washed three times with PBS for 3 min each, blocked with 0.5% bovine serum albumin (A1080; Solarbio, Beijing, China) in PBS for 30 min, and washed again three times with PBS. Primary antibodies against hTERT (1 : 100, NB100‐317SS; Novus Biologicals, Littleton, CO, USA), E‐cadherin (1 : 50, MAB43853; Bio‐Swamp), and vimentin (1 : 50, PAB40605; Bio‐Swamp) were added, and the sections were incubated overnight at 4 °C in a humidified chamber. After three washes with PBS for 5 min each, secondary antibodies from the MaxVision™ HRP‐Polymer anti‐Mouse/Rabbit IHC Kit (KIT‐5020; Maxim, Fuzhou, China) were added and the sections were incubated at room temperature for 30 min. Diaminobenzidine staining solution was added to the sections, and when color change was detected, the solution was removed with tap water. Counterstaining was performed using hematoxylin for 3 min and the sections were washed with tap water for 10 min, followed by dehydration using a series of EtOH with increasing concentration (75%, 85%, 95%, and 100%) for 5 min at each concentration. The sections were immersed in xylene, sealed in neutral balsam mounting medium, and imaged using an optical microscope. Image analysis was performed using imagepro plus (Media Cybernetics, Rockville, MD, USA), and positive areas of staining are expressed as the relative mean integrated optical density (IOD).

The article "Exosomal miR‐1255b‐5p targets human telomerase reverse transcriptase in colorectal cancer cells to suppress epithelial‐to‐mesenchymal transition" was retracted in 2023. Reasons: duplicated images; original data or images not available.

### 2.16 Statistical analysis

All data represent the mean ± SD of three biological replicates (*n* = 3) for *in vitro* assays and 10 biological replicates (*n* = 10) for *in vivo* studies. The paired‐sample *t*‐test was performed to compare differences between two groups, and one‐way analysis of variance (ANOVA) was conducted to compare differences between more than two groups, followed by Tukey's *post hoc* test. Chi‐square test and logistic regression analysis were applied to analyze the correlation between exosomal miR‐1255b‐5p expression and clinicopathological status. A *P* value of < 0.05 indicates the difference was statistically significant.

## 3 Results

### 3.1 Selection of miRNA from clinical samples and characterization of exosomes

From preliminary bioinformatics screening (dataset GSE39833), we identified three miRNAs with binding sites to the 3′UTR of hTERT (miR‐1182, one binding site; miR‐1255b‐5p, three binding sites; miR‐197‐3p, two binding sites). We detected the relative expression of these three miRNAs in exosomes isolated from the serum of clinical CRC patients and healthy individuals (Fig. 1A–C) and found that the levels of both miR‐1255b‐5p and miR‐197‐3p were significantly lower in CRC patients than in healthy individuals. The successful isolation of exosomes from clinical serum samples was validated by TEM (Fig. 1D) and western blot of exosomal markers CD63, CD81, and TSG101 (Fig. 1E,F), which showed that these markers were almost exclusively expressed in exosomes and absent in the supernatant. Given the overall expression trend and the number of binding sites of the miRNAs to the hTERT gene, we chose to use miR‐1255b‐5p in the subsequent studies as it appears to be an interesting target to investigate.

The article "Exosomal miR‐1255b‐5p targets human telomerase reverse transcriptase in colorectal cancer cells to suppress epithelial‐to‐mesenchymal transition" was retracted in 2023. Reasons: duplicated images; original data or images not available.

**Fig. 1:** Identification of CRC‐related miRNAs and exosomes in clinical serum samples. Expression of (A) miR‐1182, (B) miR‐1255b‐5p, and (C) miR‐197‐3p in exosomes isolated from clinical serum samples of CRC patients and healthy individuals. (D) TEM observation of exosomes isolated from clinical serum samples. Scale bar = 500 nm. (E) Western blot identification and (F) quantification of exosomal markers CD63, CD81, and TSG101 in the isolated exosomes and supernatants. Expression of miR‐1255b‐5p in (G) CRC cell lines (SW480, HCT116, LOVO, and HT29) and normal colon cells (FHC), as well as in (H) exosomes derived from the corresponding cell lines. (I) mRNA expression of hTERT in CRC cell lines and normal colon cells. (J) Western blot identification and (K) quantification of hTERT protein expression in CRC cell lines and normal colon cells. Statistical analysis was carried out using ANOVA. The data are expressed as the mean ± SD (*n* = 3 biological repeats); *P < 0.05, ns = not significant at *P* = 0.05.

To determine the correlation between exosomal miR‐1255b‐5p expression and CRC in a clinical setting, we measured the clinicopathological parameters of CRC patients via single‐factor (Table 1) and multivariate analysis (Table 2). Among the tested subjects, single‐factor analysis revealed a significant correlation between miR‐1255b‐5p expression and tumor stage, perineural invasion (PNI), lymphovascular invasion (LVI), and the levels of carcinoembryonic antigen (CEA) and carbohydrate antigen 19–9 (CA 19‐9; *P* < 0.05). In the case of multivariate analysis, miR‐1255b‐5p expression was correlated with tumor stage and CA 19‐9 levels (*P* < 0.05). These data indicated that miR‐1255b‐5p is strongly linked to tumor stage (III and IV) and CA 19‐9 level (≥ 37 U·mL^−1^) and revealed the negative correlation between exosomal miR‐1255b‐5p and CRC progression.

**Table 1:** Single‐factor analysis of the correlation between exosomal miR‐1255b‐5p expression and clinicopathologic parameters. Boldface indicates *P* < 0.05.

Parameters	*n* (%)	Exosomal miR‐1255b‐5p expression		
		Low	High	*P*
Age, year				
< 60	25 (35.7)	15	10	0.108
≥ 60	45 (64.3)	18	27	
Gender				
Male	40 (57.1)	16	24	0.167
Female	30 (42.9)	17	13	
Tumor site				
Colon	34 (48.6)	16	18	0.989
Rectal	36 (51.4)	17	19	
Tumor stage^a^				
I–II	36 (51.4)	5	31	**< 0.001**
III–IV	34 (48.6)	28	6	
Tumor size, cm				
< 5	33 (47.1)	21	12	0.088
≥ 5	37 (52.9)	16	21	
Tumor grade				
Poor	11 (15.7)	6	5	0.592
Moderate/good	59 (84.3)	27	32	
PNI				
Absence	50 (71.4)	17	33	**< 0.001**
Presence	20 (28.6)	16	4	
LVI				
Absence	44 (62.9)	13	31	**< 0.001**
Presence	26 (37.1)	20	6	
CEA, ng·mL^−1^				
< 5	46 (65.7)	17	29	**0.018**
≥ 5	24 (34.3)	16	8	
CA 19–9, U·mL^−1^				
< 37	52 (74.3)	16	36	**< 0.001**
≥ 37	18 (25.7)	17	1	

^a^ Tumor stage was assessed based on the 8th edition of the AJCC Cancer Staging Manual.

The article "Exosomal miR‐1255b‐5p targets human telomerase reverse transcriptase in colorectal cancer cells to suppress epithelial‐to‐mesenchymal transition" was retracted in 2023. Reasons: duplicated images; original data or images not available.

**Table 2:** Multivariate analysis of the correlation between exosomal miR–1255b–5p expression and clinicopathologic parameters. CI, confidence interval; OR, odds ratio. Boldface indicates *P* < 0.05.

Parameters	*B*	*P*	OR	95% CI
PNI	–0.755	0.415	0.470	0.076–2.888
LVI	0.807	0.534	2.242	0.176–28.485
Tumor stage (III–IV)	–3.312	**0.008**	0.036	0.003–0.419
CEA ≥ 5 ng·mL^−1^	0.437	0.621	1.549	0.274–8.769
CA 19–9 ≥ 37 U·mL^−1^	–3.187	**0.018**	0.041	0.003–0.580

Then, we examined the expression of miR‐1255b‐5p in four CRC cell lines (SW480, HCT116, LOVO, and HT29) and a normal FHC, as well as in exosomes derived from these cells. Among the CRC cell lines, the level of miR‐1255b‐5p was the highest in SW480 cells and the lowest in HCT116 cells (Fig. 1G) as well as in the corresponding exosomes (Fig. 1H). We evaluated the mRNA and protein expression of hTERT in the abovementioned cell lines and found that, contrary to miR‐1255b‐5p, the mRNA (Fig. 1I) and protein (Fig. 1J,K) expression of hTERT was the lowest in SW480 cells and significantly higher in HCT116 cells (even though LOVO and HT29 showed the highest expression). Based on these observations, SW480 and HCT116 cells were selected for the following experiments.

### 3.2 Hypoxia‐induced downregulation of miR‐1255b‐5p‐mediated properties are transferred via exosomal delivery

Oxygen deficiency in the tumor microenvironment has been linked to rapid tumor growth and metastasis [21]. To investigate whether oxygen deficiency affects the expression of miR‐1255b‐5p and its target gene, we cultured SW480 cells (previously shown to exhibit high expression of miR‐1255b‐5p) in normoxic and hypoxic conditions (denoted as SW480/Norm and SW480/Hyp, respectively). qRT‐PCR (Fig. 2A) revealed that the expression of miR‐1255b‐5p was significantly higher in SW480/Norm than that in SW480/Hyp, whereas hTERT showed the opposite trend. The gene expression of HIF‐1α, a marker of hypoxia, was drastically upregulated by hypoxic conditions, as expected. The protein expression of hTERT and HIF‐1α was consistent with that of mRNA expression (Fig. 2B). We then isolated exosomes from SW480/Norm and SW480/Hyp (denoted as SW480/Norm‐Exo and SW480/Hyp‐Exo, respectively) and confirmed their successful isolation using TEM (Fig. 2C) and western blot identification of exosomal markers (Fig. 2D). We further confirmed that the expression of miR‐1255b‐5p was significantly lower in exosomes isolated in a hypoxic environment compared to that in normoxic exosomes (Fig. 2E). This signifies that the isolated exosomes carried miR‐1255b‐5p and that the change in oxygen condition elicited simultaneous changes in exosomal cargo.

The article "Exosomal miR‐1255b‐5p targets human telomerase reverse transcriptase in colorectal cancer cells to suppress epithelial‐to‐mesenchymal transition" was retracted in 2023. Reasons: duplicated images; original data or images not available.

**Fig. 2:** Effect of hypoxia on miR‐1255b‐5p expression and transfer of miR‐1255b‐5p‐containing exosomes between CRC cells. (A) qRT‐PCR analysis of miR‐1255b‐5p expression and mRNA expression of hTERT and HIF‐1α in SW480 cells cultured in normoxic (SW480/Norm) and hypoxic (SW480/Hyp) conditions. (B) Western blot and quantification of the protein expression of hTERT and HIF‐1α in SW480 cells cultured in normoxic and hypoxic conditions. (C) TEM observation of exosomes derived from SW480/Norm and SW480/Hyp. Scale bar = 500 nm. (D) Western blot identification of exosomal markers CD63, CD81, and TSG101 and the endogenous control GAPDH in exosomes derived from SW480/Norm or SW480/Hyp and in cell lysates. (E) Expression of miR‐1255b‐5p in exosomes derived from SW480/Norm and SW480/Hyp. (F) Fluorescence imaging of PKH67‐stained exosomes endocytosed by HCT116 cells for 2, 24, and 48 h. Green fluorescence indicates PKH67 staining and blue fluorescence represents cell nuclei. Scale bar = 50 μm. (G) Scratch assay performed in HCT116 cells cultured with SW480/Norm‐Exo or SW480/Hyp‐Exo for 0, 24, or 48 h. Representative image was chosen among three replicates. Gap width was measured using imagej. Scale bar = 200 μm. (H) CCK‐8 assay of HCT116 cell proliferation after 24 or 48 h of culture with SW480/Norm‐Exo or SW480/Hyp‐Exo. (I) Transwell assay and (J) quantification of HCT116 cell invasion after 24 or 48 h of culture with SW480/Norm‐Exo or SW480/Hyp‐Exo. Scale bar = 100 μm. (K) miR‐1255b‐5p expression and mRNA expression of hTERT, E‐cadherin, and vimentin in HCT116 cells cultured with SW480/Norm‐Exo or SW480/Hyp‐Exo. (L) Western blot and quantification of the expression of hTERT and proteins associated with EMT (E‐cadherin, vimentin, Wnt1, and β‐catenin) in HCT116 cells cultured with SW480/Norm‐Exo or SW480/Hyp‐Exo. (M) Telomerase content and (N) telomere length in HCT116 cells cultured with SW480/Norm‐Exo or SW480/Hyp‐Exo. Statistical analysis was carried out using ANOVA. The data are expressed as the mean ± SD (*n* = 3 biological repeats); *P < 0.05.

We next investigated whether SW480‐derived exosomes could deliver and release their cargo into HCT116 cells, which are deficient in miR‐1255b‐5p. HCT116 cells were cultured with exosomes from SW480/Norm or SW480/Hyp, and exosomal uptake was evaluated over a period of 48 h using PKH67 labeling (Fig. 2F). In both cases, the bright green fluorescence confirmed that exosomes were endocytosed by HCT116 cells. A series of experiments were performed to evaluate the effect of normoxic and hypoxic exosomes on the biological behavior of HCT116, such as proliferation, survival, invasion, and protein expression. Scratch assay (Fig. 2G) demonstrated that within 48 h, HCT116 cells cultured with SW480/Hyp‐Exo closed the scratched gap (~ 79% closure) much more effectively than did control cells (~ 67% closure) or those cultured with SW480/Norm‐Exo (~ 65% closure). CCK‐8 assay (Fig. 2H) revealed that compared to control HCT116 cells, those treated with exosomes exhibited significantly higher degree of proliferation, but the hypoxic exosomes exerted a much more prominent effect. These results are supported by EdU staining for proliferation (Fig. S1a) and flow cytometry for apoptosis (Fig. S1b). Furthermore, Transwell assay illustrated that SW480/Hyp‐Exo enhanced the invasive ability of HCT116 cells compared to SW480/Norm‐Exo (Fig. 2I,J).

The article "Exosomal miR‐1255b‐5p targets human telomerase reverse transcriptase in colorectal cancer cells to suppress epithelial‐to‐mesenchymal transition" was retracted in 2023. Reasons: duplicated images; original data or images not available.

To elucidate the possible regulation of EMT by SW480‐derived exosomes, we evaluated the expression of main proteins involved in EMT (E‐cadherin and vimentin) and changes in the Wnt/β‐catenin pathway. First, qRT‐PCR (Fig. 2K) revealed that normoxic exosomes upregulated miR‐1255b‐5p and downregulated the mRNA expression of hTERT in HCT116 cells. Meanwhile, the mRNA expression of anti‐EMT E‐cadherin was upregulated and pro‐EMT vimentin was downregulated. Hypoxic exosomes showed an opposite trend as that of normoxic exosomes in all cases. Next, the protein expression of hTERT, E‐cadherin, vimentin, Wnt1, and β‐catenin was measured (Fig. 2L). As anticipated, normoxic exosomes reduced the protein expression of hTERT and the pro‐EMT vimentin, Wnt1, and β‐catenin while elevating that of the anti‐EMT E‐cadherin. Again, hypoxic exosomes showed an opposite trend as that of normoxic exosomes in all cases. As a validation of hTERT function, we examined the effect of exosomes on telomerase content (Fig. 2M) and telomere length (Fig. 2N) in HCT116 cells cultured with normoxic or hypoxic SW480‐derived exosomes. There was no significant difference in telomerase content, but the telomere length was significantly increased when HCT116 cells were cultured with hypoxic exosomes than that in cells cultured with normoxic exosomes.

Collectively, the results demonstrated that exosomal content derived from SW480 cells, which included miR‐1255b‐5p, was delivered to HCT116 cells, but the function of the delivered exosomes were influenced by hypoxic microenvironmental conditions. While normoxic exosomes inhibited the growth of CRC cells possibly via miR‐1255b‐5p delivery, oxygen deficiency instead conferred tumorigenic and metastatic traits to HCT116 cells via exosomal transfer. This occurs via the upregulation of hTERT, promotion of pro‐EMT factors, and telomere lengthening.

The article "Exosomal miR‐1255b‐5p targets human telomerase reverse transcriptase in colorectal cancer cells to suppress epithelial‐to‐mesenchymal transition" was retracted in 2023. Reasons: duplicated images; original data or images not available.

### 3.3 miR‐1255b‐5p regulated EMT of HCT116 cells via exosomal delivery

Having demonstrated the important tumor‐suppressing role of miR‐1255b‐5p in CRC cells, we overexpressed or silenced miR‐1255b‐5p by transfecting hypoxic SW480 cells with miR‐1255b‐5p mimics or inhibitors. The transfection efficiency was confirmed by detecting the expression of miR‐1255b‐5p in hypoxic SW480 cells subjected to miR‐1255b‐5p inhibitor (inh) or mimic (mim) transfection, as well as their corresponding NC (Fig. 3A). Exosomes derived from the transfected SW480 cells showed the same tendency as the host cells (Fig. 3B), indicating that transfection of mimics or inhibitors affected exosomal miR‐1255b‐5p. HCT116 cells, which are deficient in miR‐1255b‐5p, were then cultured with exosomes isolated from nontransfected hypoxic SW480 cells (SW480/Hyp‐Exo) or those transfected with miR‐1255b‐5p inhibitors (SW480/Hyp/inh‐Exo) or mimics (SW480/Hyp/mim‐Exo), and the exosomal uptake efficiency was confirmed by PKH67 staining (Fig. 3B). Scratch assay (Fig. 3C) demonstrated that within 48 h, HCT116 cells cultured with SW480/inh/Hyp‐Exo closed the scratched gap (~ 61% closure) much more effectively than those cultured with SW480/Hyp‐Exo (~ 47% closure) or SW480/mim/Hyp‐Exo (~ 27% closure). This revealed that exosomal miR‐1255b‐5p inhibition enhanced the proliferative and migratory ability of HCT116 cells, whereas overexpression of miR‐1255b‐5p had the opposite effect, and these results are supported by CCK‐8 assay (Fig. 3D), EdU staining (Fig. S2a), and flow cytometry (Fig. S2b). HCT116 cell invasion showed the same trend, as miR‐1255b‐5p inh‐transfected SW480 cells produced exosomes that promoted HCT116 cell invasion, while those derived from miR‐1255b‐5p mimic‐transfected SW480 cells suppressed HCT116 cell invasion (Fig. 3E,F).

**Fig. 3:** Effect of miR‐1255b‐5p overexpression and inhibition on CRC behavior via delivery of miR‐1255b‐5p‐containing exosomes. (A) qRT‐PCR of the transfection efficiency of miR‐1255b‐5p inhibitors (inh) and mimics (mim) as well as the corresponding NC (inh) and NC (mim), respectively. miR‐1255b‐5p expression was measured in transfected SW480 cells and isolated exosomes. (B) Fluorescence imaging of PKH67‐stained exosomes endocytosed by HCT116 cells for 2, 24, and 48 h. Green fluorescence indicates PKH67 staining and blue fluorescence represent cell nuclei. Scale bar = 50 μm. (C) Scratch assay performed in HCT116 cells cultured with SW480/Hyp/inh‐Exo or SW480/Hyp/mim‐Exo for 0, 24, or 48 h. Representative image was chosen among three replicates. Gap width was measured using imagej. Scale bar = 200 μm. (D) CCK‐8 assay of HCT116 cell proliferation after 24 or 48 h of culture with SW480/Hyp/inh‐Exo or SW480/Hyp/mim‐Exo. (E) Transwell assay and (F) quantification of HCT116 cell invasion after 24 or 48 h of culture with SW480/Hyp/inh‐Exo or SW480/Hyp/mim‐Exo. Scale bar = 100 μm. (G) miR‐1255b‐5p expression and mRNA expression of hTERT, E‐cadherin, and vimentin in HCT116 cells cultured with SW480/Hyp/inh‐Exo or SW480/Hyp/mim‐Exo. (H) Western blot and (I) quantification of the expression of hTERT and proteins associated with EMT (E‐cadherin, vimentin, Wnt1, and β‐catenin) in HCT116 cells cultured with SW480/Hyp/inh‐Exo or SW480/Hyp/mim‐Exo. (J) Telomerase content and (K) telomere length in HCT116 cells cultured with SW480/Hyp/inh‐Exo or SW480/Hyp/mim‐Exo. Statistical analysis was carried out using ANOVA. The data are expressed as the mean ± SD (*n* = 3 biological repeats); *P < 0.05.

The article "Exosomal miR‐1255b‐5p targets human telomerase reverse transcriptase in colorectal cancer cells to suppress epithelial‐to‐mesenchymal transition" was retracted in 2023. Reasons: duplicated images; original data or images not available.

Next, we examined whether miR‐1255b‐5p (Fig. 3G) mimics or inhibitors regulated EMT and pathways involved therein. qRT‐PCR indicated that HCT116 cells cultured with SW480/Hyp/mim‐Exo and SW480/Hyp/inh‐Exo showed opposite tendencies between miR‐1255b‐5p and hTERT mRNA expression. In addition, overexpression of miR‐1255b‐5p upregulated the gene expression of the anti‐EMT E‐cadherin but downregulated that of the pro‐EMT vimentin, while miR‐1255b‐5p inhibitors had the opposite effect. The protein expression of hTERT, E‐cadherin, and vimentin was consistent with the results of gene expression. Moreover, activation of the Wnt/β‐catenin pathway was promoted by miR‐1255b‐5p inhibition but remarkably suppressed by miR‐1255b‐5p overexpression, as demonstrated by the protein expression of Wnt1 and β‐catenin (Fig. 3H,I). In association with hTERT, telomerase content (Fig. 3J) and telomere length (Fig. 3K) were measured. Delivery of miR‐1255b‐5p‐overexpressing exosomes resulted in significantly reduced telomere length in HCT116 cells compared to SW480/Hyp‐Exo and the negative controls NC(i) and NC(m), whereas exosomes expressing low levels of miR‐1255b‐5p greatly lengthened the telomeres of HCT116 cells.

Taken together, these observations suggest that overexpression or inhibition of miR‐1255b‐5p in host SW480 cells under hypoxic conditions resulted in the release of exosomes carrying corresponding amounts of miR‐1255b‐5p. These exosomes then exerted the corresponding effects of miR‐1255b‐5p in HCT116 cells via intercellular communication.

### 3.4 Targeting relationship between miR‐1255b‐5p and hTERT and mechanism underlying EMT regulation

We took a closer look at the potential targeting relationship between miR‐1255b‐5p and hTERT, as well as the specific role of hTERT in regulating EMT. Bioinformatic analysis has identified three binding sites between miR‐1255b‐5p and the 3′UTR of the hTERT gene (Fig. 4A) and thus, dual‐luciferase activity assay was performed to confirm binding at these sites (Fig. 4B). Having established this targeting relationship and having already shown that miR‐1255b‐5p is associated with EMT, we investigated whether hTERT was involved therein and elucidated the underlying mechanisms. To do this, we silenced hTERT via transfection of hTERT interference (si‐hTERT) vectors (with empty vectors as NC, nc‐hTERT) in both SW480 and HCT116 cells. The transfection efficiency was confirmed by the significant decrease in the mRNA expression of hTERT in both cell types upon si‐hTERT transfection (Fig. 4C). The expression of EMT‐associated proteins was then detected in the transfected CRC cells (Fig. 4D). In both SW480 (Fig. 4E) and HCT116 (Fig. 4F) cells, hTERT interference significantly upregulated the protein expression of E‐cadherin but downregulated that of vimentin, Wnt1, and β‐catenin. This signifies the positive correlation between hTERT and EMT, as the inhibition of hTERT suppressed pro‐EMT protein expression. In terms of cell invasion (Fig. 4G), SW480 (Fig. 4H) and HCT116 (Fig. 4I) cells transfected with si‐hTERT showed a decrease in cell count after 48 h, indicating that si‐hTERT may suppress the metastatic ability of CRC cells via the inhibition of EMT.

The article "Exosomal miR‐1255b‐5p targets human telomerase reverse transcriptase in colorectal cancer cells to suppress epithelial‐to‐mesenchymal transition" was retracted in 2023. Reasons: duplicated images; original data or images not available.

**Fig. 4:** Verification of targeting relationship between miR‐1255b‐5p and hTERT and function of hTERT in EMT. (A) Binding sites between miR‐1255b‐5p and the 3′UTR of the hTERT promoter at 1278–1284 bp, 1309–1315 bp, and 1420–1427 bp. (B) Dual‐luciferase activity assay of the binding between miR‐1255b‐5p and the 3′UTR of hTERT. (C) qRT‐PCR of the mRNA expression of hTERT in SW480 and HCT116 transfected with hTERT interference (si‐hTERT) vectors, with empty vectors (nc‐hTERT) as a NCs. (D) Western blot of the expression of hTERT and proteins associated with EMT (E‐cadherin, vimentin, Wnt1, and β‐catenin) in SW480 and HCT116 cells transfected with nc‐hTERT or si‐hTERT. Quantification of EMT‐associated protein expression in transfected (E) SW480 and (F) HCT116 cells. (G) Transwell assay of SW480 and HCT116 cell invasion after transfection with nc‐hTERT or si‐hTERT. Scale bar = 100 μm. Quantification of the number of invasive (H) SW480 and (I) HCT116 cells. (J) GST pull‐down assay demonstrating the interaction between hTERT and BRG1, in HCT116 cells cultured with exosomes from inh/mim‐transfected hypoxic SW480 cells. Statistical analysis was carried out using ANOVA. The data are expressed as the mean ± SD (*n* = 3 biological repeats); *P < 0.05, ns = not significant at *P* = 0.05.

The article "Exosomal miR‐1255b‐5p targets human telomerase reverse transcriptase in colorectal cancer cells to suppress epithelial‐to‐mesenchymal transition" was retracted in 2023. Reasons: duplicated images; original data or images not available.

We suspected that the way through which hTERT mediates EMT is related to reported mechanisms that involve binding of hTERT to BRG1. We thus performed a GST pull‐down assay to validate the relationship between hTERT and BRG1 (Fig. 4J), which is required for the co‐binding of hTERT and ZEB1 to the CDH1 gene encoding E‐cadherin [16]. Herein, we again cultured HCT116 cells with exosomes derived from hypoxic SW480 cells transfected with miR‐1255b‐5p mimics or inhibitors. Among the five groups, the addition of SW480/inh/Hyp‐Exo induced a remarkable increase in the amount of BRG1 pulled down by the assay. This result indicates that miR‐1255b‐5p inhibition, which effectively upregulated hTERT as previously shown, significantly elevated the protein expression of BRG1. As the pull‐down of BRG1 is related to its binding to GST‐conjugated hTERT, we hypothesize here that the increase in hTERT induced by miR‐1255b‐5p inhibition could be a cause of BRG1 upregulation. In other words, hTERT bound to BRG1, and the two were simultaneously upregulated by miR‐1255b‐5p inhibition.

### 3.5 Rescue assays to determine the specific mechanism of hTERT suppression by miR‐1255b‐5p

On the premise that SW480 and HCT116 cells express high and low levels of miR‐1255b‐5p, respectively, we performed rescue experiments to determine that the observed effects of miR‐1255b‐5p and hTERT were indeed due to the targeting relationship between the two. In SW480 cells, miR‐1255b‐5p expression was silenced by inhibitors, and this was accompanied by the transfection of si‐hTERT (Fig. 5A). The opposite was performed in HCT116 cells, wherein miR‐1255b‐5p was overexpressed using mimics, with or without the overexpression of hTERT (Fig. 5B). Essentially, we examined whether hTERT interference or overexpression opposed the effects of miR‐1255b‐5p inhibition or overexpression, respectively, on biological behavior and EMT. As revealed in Fig. 5C, SW480 cells transfected with miR‐1255b‐5p inhibitors showed increased proliferation (consistent with Fig. 3D), but this was counteracted by hTERT interference. On the other hand, HCT116 cells transfected with miR‐1255b‐5p mimics showed a decrease in proliferation (Fig. 5D), which was consistent with the result of Fig. 3D. In turn, hTERT overexpression counteracted the effect of miR‐1255b‐5p mimics by increasing the proliferation of HCT116 cells.

**Fig. 5:** Verification of the effect and mechanism of hTERT on EMT via rescue experiments. miR‐1255b‐5p expression and mRNA expression of hTERT in (A) SW480 cells transfected with miR‐1255b‐5p inhibitors and si‐hTERT and in (B) HCT116 cells transfected with miR‐1255b‐5p mimics and hTERT overexpression vectors. CCK‐8 assay of the proliferation of (C) SW480 cells transfected with miR‐1255b‐5p inhibitors and si‐hTERT and of (D) HCT116 cells transfected with miR‐1255b‐5p mimics and hTERT overexpression vectors. Western blot and quantification of hTERT and EMT‐associated proteins (E‐cadherin, vimentin, Wnt1, and β‐catenin) in (E) SW480 cells transfected with miR‐1255b‐5p inhibitors and si‐hTERT and of (F) HCT116 cells transfected with miR‐1255b‐5p mimics and hTERT overexpression vectors. Transwell assay and quantification of the number of invasive (G) SW480 cells transfected with miR‐1255b‐5p inhibitors and si‐hTERT and of (H) HCT116 cells transfected with miR‐1255b‐5p mimics and hTERT overexpression vectors. Scale bar = 100 μm. (I) Decay curve showing the expression of hTERT mRNA in HCT116 transfected with miR‐1255b‐5p mimics or NC. Statistical analysis was carried out using ANOVA. The data are expressed as the mean ± SD (*n* = 3 biological repeats); *P < 0.05.

The article "Exosomal miR‐1255b‐5p targets human telomerase reverse transcriptase in colorectal cancer cells to suppress epithelial‐to‐mesenchymal transition" was retracted in 2023. Reasons: duplicated images; original data or images not available.

In addition, the protein expression of EMT‐associated factors was detected in SW480 (Fig. 5E) and HCT116 (Fig. 5F) cells. Inhibition of miR‐1255b‐5p decreased the protein expression of E‐cadherin and increased hTERT, vimentin, Wnt1, and β‐catenin expression in SW480 cells, whereas miR‐1255b‐5p overexpression induced the opposite phenomenon in HCT116 cells. Upon hTERT interference or overexpression, respectively, the effect of miR‐1255b‐5p inhibitors/mimics was counteracted. Transwell invasion assay showed the same trend, wherein the increase or decrease in SW480 or HCT116 cells by miR‐1255b‐5p inhibitors or mimics was opposed by si‐hTERT or hTERT overexpression, respectively (Fig. 5G,H).

It has been suggested that miRNAs suppress the expression of their targets via two forms of interaction. They either bind directly to the target mRNA to disrupt its stability or degrade the target protein post‐transcriptionally [22]. The former mode is manifested by a gradual decrease in target mRNA over time compared to the nonbinding circumstance, whereas the latter does not induce changes at the transcription level. To determine the mode through which miR‐1255b‐5p suppresses the activity of its target hTERT, we cultured HCT116 cells with miR‐1255b‐5p mimics or NC and measured the mRNA expression of hTERT at various time points (0, 2, 4, 8, and 16 h) by qRT‐PCR. The electrophoretic bands and mRNA decay curve in Fig. 5I illustrate that with the NC, hTERT mRNA exhibits a gradual decrease with a decay half‐life of 4.67 h. This is due to the fact that in normal physiological circumstances, mRNA is translated into protein gradually. However, our observations of miR‐1255b‐5p mimic transfection revealed that the overall hTERT mRNA level was lower than the NC at all time points of detection, with a decay half‐life of 1.42 h. This suggests that miR‐1255b‐5p greatly affected the stability of hTERT mRNA, supporting the mode of direct miRNA‐mRNA binding in the mechanism of target suppression.

The article "Exosomal miR‐1255b‐5p targets human telomerase reverse transcriptase in colorectal cancer cells to suppress epithelial‐to‐mesenchymal transition" was retracted in 2023. Reasons: duplicated images; original data or images not available.

### 3.6 **Effect of miR‐1255b‐5p‐carrying exosomes on EMT, CRC progression, and liver metastasis** *in vivo*

The aforementioned findings regarding the association between miR‐1255b‐5p and hTERT in relation to EMT were validated in an *in vivo* nude mouse model of xenografted CRC tumor. Exosomes containing various amounts of miR‐1255b‐5p (induced by mimic or inh transfection) were injected in nude mice subjected to CRC tumor xenografting (Fig. 6A). At the end of 20 days, the volume (Fig. 6B) and weight (Fig. 6C) of the tumors in mice injected with SW480/Hyp/inh‐Exo (exosomes derived from hypoxic SW480 cells transfected with miR‐1255b‐5p inhibitors) were significantly higher than those of mice in the other groups. This observation indicates that the inhibition of miR‐1255b‐5p, which we previously identified as antitumorigenic, promoted tumor growth. Detection of the mRNA (Fig. 6D) and protein expression of hTERT and EMT‐associated factors in tumor tissues (Fig. 6E,F) revealed the same trend as that shown in the *in vitro* studies. Finally, we examined the morphology of tumor (Fig. 6G) and liver (Fig. 6H) tissues to assess the progression of CRC and liver metastasis in the experimental animals by H&E staining. Immunohistochemical staining also revealed that the expression of hTERT, E‐cadherin, and vimentin was consistent with the trend shown in the *in vitro* experiments and with that of *in vivo* western blot (Fig. 6I). Specifically, miR‐1255b‐5p overexpression resulted in decreased expression of hTERT and vimentin and increased expression of E‐cadherin, which are indicative of EMT, in both tumor and liver tissues. These results confirmed that exosomes derived from hypoxic SW480 cells had varying effects on colorectal tumor progression and liver metastasis depending on the amount of miR‐1255b‐5p carried by the exosomes.

**Fig. 6:** Effect of miR‐1255b‐5p‐containing exosomes on CRC progression and liver metastasis in *in vivo* xenograft model of CRC. (A) Photographs of colorectal tumors extracted from xenografted nude mice that were treated with exosomes derived from hypoxic SW480 cells containing varying amounts of miR‐1255b‐5p. Tumors were extracted after the mice were sacrificed on day 20. (B) Tumor growth curve during the 20‐day experimental period. (C) Tumor weight at day 20, after the mice were sacrificed and tumors were extracted. (D) miR‐1255b‐5p expression and mRNA expression of hTERT, E‐cadherin, and vimentin in tumor tissues extracted from mice subjected to exosome treatment. (E) Western blot and (F) quantification of hTERT and EMT‐associated proteins (E‐cadherin, vimentin, Wnt1, and β‐catenin) in tumor tissues extracted from mice subjected to exosome treatment. H&E staining of tissue morphology and immunohistochemical staining of hTERT, E‐cadherin, and vimentin protein expression in (G) colorectal tumor tissues and (H) liver tissues. Scale bar = 50 μm. (I) Quantification of positive areas of staining for hTERT, E‐cadherin, and vimentin. The data represent the relative mean IOD measured by imagepro plus. Statistical analysis was carried out using ANOVA. The data are expressed as the mean ± SD (*n* = 10 biological repeats); *P < 0.05.

The article "Exosomal miR‐1255b‐5p targets human telomerase reverse transcriptase in colorectal cancer cells to suppress epithelial‐to‐mesenchymal transition" was retracted in 2023. Reasons: duplicated images; original data or images not available.

## 4 Discussion

Exosomes produced in the tumor microenvironment interact with target cells in various ways. They can directly stimulate ligands that are expressed on the target cell membrane or affect the recipient cell via endocytosis [23]. Furthermore, genetic information contained within the exosomes, such as miRNAs and mRNA, can be transferred between tumor and target cells. As a consequence, disruptions in the tumor microenvironment induce corresponding changes in exosomal content and affect the production and secretion of exosomes. Among the factors that alter the tumor microenvironment, hypoxia plays a substantial role in malignant progression in ways such as enhancing metastatic potential and conferring resistance against anticancer therapy [24]. Particularly in CRC, hypoxia promotes EMT‐induced migration and metastasis, a process involving factors such as USP47 and SIRT1 [25, 26].

The effect of hypoxia on telomerase activity and telomere elongation, which is critical in cancer onset and progression [27], has been well established. Hypoxia reportedly not only triggers the activation of the hTERT promoter, but also upregulates the expression of endogenous hTERT, and these phenomena are mediated by HIF‐1 [17]. hTERT activation in turn enables telomere length to be maintained, thereby allowing tumor cells to grow indefinitely. Complementary effects associated with HIF metabolic reprogramming may also be implicated in cancer cell metabolism. For example, HIF‐regulated aerobic glycolysis (Warburg effect) may lead to vascular endothelial growth factor‐dependent tumor angiogenesis, which is conducive to tumor growth [28]. HIF‐mediated signaling in turn is tightly linked to pathways that promote EMT, invasion, and metastasis, among other tumor‐related biological processes [29]. Moreover, large‐scale studies of hypoxic tumors have been carried out to identify dysregulated miRNAs associated with hypoxia [30]. Some commonly known hypoxia‐related miRNAs include miR‐210 [31], miR‐133a [32], and miR‐590‐5p [33]. Our study identified miR‐1255b‐5p as a tumor‐suppressing miRNA that exhibited altered expression in hypoxic conditions compared to that in a normoxic environment. Reports on the characteristics and functions of miR‐1255b‐5p, however, remain scarce, especially with regards to its role in CRC and EMT.

The article "Exosomal miR‐1255b‐5p targets human telomerase reverse transcriptase in colorectal cancer cells to suppress epithelial‐to‐mesenchymal transition" was retracted in 2023. Reasons: duplicated images; original data or images not available.

It has been proposed that miRNAs suppress the expression of their target genes by either enhancing mRNA degradation or promoting translational repression. In particular, miRNAs function by interacting with an RNA‐induced silencing complex (RISC) to mediate gene targeting [22]. In mammalian cells, miRNAs can promote mRNA degradation via target slicing. This requires the presence of a slicer, known as Argonaute or Ago [34], as well as highly precise complementarity between the miRNA and its target mRNA. Degradation is mediated by exonucleases and occurs when the miRNA breaks the reading frame of the encoded protein, resulting in target mRNA hydrolysis [35]. Meanwhile, translation repression does not require perfect complementarity and proceeds through the interaction of miRNAs with Ago. Even in the same organism, different types of Ago can function via different mechanisms to control gene suppression. In Drosophila, Ago1 but not Ago2 induces target mRNA deadenylation. On the other hand, Ago2 forms a complex with the RISC to inhibit protein interaction between the eukaryotic initiation factors 4E and 4G, effectively blocking translation initiation [36].

Herein, we propose that the mechanism through which miR‐1255b‐5p targets the expression of hTERT is through mRNA degradation, as demonstrated by the faster decay in mRNA expression in cells treated with miR‐1255b‐5p compared to that in control cells. The inhibition of hTERT has crucial implications in the process of EMT in tumor development and metastasis. In a study by Qin *et al*. [15], the process through which hTERT affects EMT was demonstrated. Specifically, the interaction between hTERT and ZEB1 enables the formation of a complex that inhibits E‐cadherin expression by binding to the 1954–1959 bp region of the E‐cadherin promoter [16]. In addition, the recruitment of BRG1, a component of the SWI/SNF chromatin‐remodeling complex [37], is required in this process. E‐cadherin is an important protein that signifies the integrity of cell‐cell junctions. During EMT initiation, cell–cell junctions (including tight junctions, adherens junctions, and gap junctions) are dissembled and degraded, resulting in the cleavage of E‐cadherin [38]. Consequently, the loss of E‐cadherin expression is a defining characteristic of EMT, whereby cell migration and invasion are promoted and metastatic potential is enhanced. In our case, hTERT expression is promoted by miR‐1255b‐5p inhibition, which triggers the formation of the hTERT‐ZEB1 complex. As a consequence, this complex binds to the E‐cadherin promoter, and E‐cadherin is downregulated while EMT is promoted, as evidenced both *in vitro* and *in vivo* in our study.

The article "Exosomal miR‐1255b‐5p targets human telomerase reverse transcriptase in colorectal cancer cells to suppress epithelial‐to‐mesenchymal transition" was retracted in 2023. Reasons: duplicated images; original data or images not available.

Furthermore, the Wnt/β‐catenin signaling pathway, which has been recognized as an important target in anticancer therapies [39], participates in EMT and the maintenance of telomerase activity. During EMT, cells lose their epithelial phenotype and transform into mesenchymal cell types, a process that results in the loss of cell‐cell adhesion and enhanced motility. The E‐cadherin/β‐catenin complex is the main regulator of epithelial integrity. Destabilization of cell–cell contact leads to the degradation of the E‐cadherin/β‐catenin junction, whereby E‐cadherin is downregulated and β‐catenin is translocated from the cytoplasm to the cell nucleus [40]. There, β‐catenin interacts with a series of transcription factors in the T‐cell factor/lymphoid enhancer factor family to regulate processes such as cell adhesion and tumor development [41]. β‐catenin is also a key effector of canonical Wnt signaling, the regulation of which mediates changes in the expression of various genes associated with EMT. Among these EMT‐associated factors, the relative levels of E‐cadherin and vimentin commonly serve as markers of EMT progression. Interestingly, a vital link has been established between telomerase activity and Wnt/β‐catenin signaling in cancer cells [42]. In particular, TCF4 forms a complex with β‐catenin in the nucleus that activates the hTERT promoter to enhance telomerase activity [43]. hTERT and β‐catenin have also been found to be co‐expressed at the invasive front of CRC [44], suggesting the co‐regulatory relationship between the two. Our results showing that hTERT silencing inhibited the expression of genes and proteins associated with EMT (E‐cadherin and vimentin) and Wnt/β‐catenin signaling (Wnt1 and β‐catenin) are consistent with the literature. The targeting relationship between miR‐1255b‐5p and hTERT thus reveals that miR‐1255b‐5p had an inhibitory effect on EMT and Wnt/β‐catenin signaling, further confirming its tumor‐suppressing role in CRC cells. Moreover, clinical research indicated that the expression of the exosomal miRNA‐1255b‐5p was significantly associated with tumor stage and CA 19‐9 levels in CRC patients. The later the tumor stage, the lower the exosomal miR‐1255b‐5p expression level. Exosomal miR‐1255b‐5p is negatively correlated with CRC progression.

The article "Exosomal miR‐1255b‐5p targets human telomerase reverse transcriptase in colorectal cancer cells to suppress epithelial‐to‐mesenchymal transition" was retracted in 2023. Reasons: duplicated images; original data or images not available.

## 5 Conclusions

Through this study, we revealed the critical tumor‐suppressing role of miR‐1255b‐5p in CRC through the inhibition of EMT, and we showed that miR‐1255b‐5p could be transmitted via exosomal delivery between CRC cells with different miR‐1255b‐5p expression profiles. In this way, CRC‐derived exosomes are horizontally transferred between CRC cells as a form of cellular crosstalk. In physiological conditions, microenvironmental changes such as hypoxia cause a decline in the level of miR‐1255b‐5p, correspondingly lowering the miR‐1255b‐5p content in CRC‐derived exosomes. Importantly, we confirmed the targeting relationship between miR‐1255b‐5p and hTERT and demonstrated the mechanism through which miR‐1255b‐5p suppresses EMT, which involves the disruption of telomerase stability and inhibition of Wnt/β‐catenin pathway activation through hTERT inhibition. More importantly, hypoxic microenvironments play an important role in tumor progression. Hypoxia directly affected exosomal miR‐1255b‐5p content, increasing hTERT expression, which promoted EMT and enhanced telomerase content and stability. The findings presented here provide a clear picture of some of the factors involved in EMT regulation in CRC cells and contribute to the future development of anticancer therapies by suggesting hTERT and telomere activity as therapeutic targets in CRC treatment.

## Conflict of interest

The authors declare no conflict of interest.

## Author contributions

XZ performed most of the experiments and wrote the manuscript. JB assisted in the key experiments of the study. ZZ assisted in data collection and analysis. HY was involved in handling the animal experiments. LL assisted in the revision of the manuscript. QW was involved in handling the animal experiments. FC and XY assisted in the *in vitro* experiments. YZ designed the study and obtained funding to support this research.

## Ethics approval and consent to participate

All animal experiments were performed in accordance with the Guidelines for Animal Care and Use of the Model Animal Research Institute at Wuhan Myhalic Biotechnology Co., Ltd., and have been approved by the institutional review board (approval number HLK‐20181031‐01).

## Consent for publication

All clinical samples were collected with informed consent from the patients, and all related procedures were performed with the approval of the internal review and ethics boards of Zhongnan Hospital of Wuhan University.

The article "Exosomal miR‐1255b‐5p targets human telomerase reverse transcriptase in colorectal cancer cells to suppress epithelial‐to‐mesenchymal transition" was retracted in 2023. Reasons: duplicated images; original data or images not available.

## Supporting information


**Data S1**. Supplementary materials.

**Fig. S1**. Effect of hypoxic exosomal delivery on the proliferation and apoptosis of HCT116 cells.

**Fig. S2**. Effect of miR‐1255b‐5p overexpression and inhibition on the proliferation and apoptosis of HCT116 cells via delivery of miR‐1255b‐5p‐containing exosomes.

**Fig. S3**. Rescue assay of miR‐1255b‐5p overexpression/inhibition and hTERT overexpression/inhibition in terms of SW480 and HCT116 cell apoptosis.

## Data Availability

The datasets used and/or analyzed during the current study are available from the corresponding author on reasonable request.
